This article has been retracted.

# Development and Optimization of Luliconazole Spanlastics to Augment the Antifungal Activity against *Candida albicans*

**DOI:** 10.3390/pharmaceutics13070977

**Published:** 2021-06-28

**Authors:** Nabil A. Alhakamy, Mohammed W. Al-Rabia, Shadab Md, Alaa Sirwi, Selwan Saud Khayat, Sahar Saad AlOtaibi, Raghad Abkar Hakami, Hadeel Al Sadoun, Basmah Medhat Eldakhakhny, Wesam H. Abdulaal, Hibah M. Aldawsari, Shaimaa M. Badr-Eldin, Mahmoud A. Elfaky

**Affiliations:** 1 Department of Pharmaceutics, Faculty of Pharmacy, King Abdulaziz University, Jeddah 21589, Saudi Arabia; nalhakamy@kau.edu.sa (N.A.A.); shaque@kau.edu.sa (S.M.); Selwankhayat@gmail.com (S.S.K.); Otaibisah@gmail.com (S.S.A.); Raghad120012@gmail.com (R.A.H.); haldosari@kau.edu.sa (H.M.A.); 2 Advanced Drug Delivery Research Group, Faculty of Pharmacy, King Abdulaziz University, Jeddah 21589, Saudi Arabia; 3 Center of Excellence for Drug Research and Pharmaceutical Industries, King Abdulaziz University, Jeddah 21589, Saudi Arabia; 4 Department of Medical Microbiology and Parasitology, Faculty of Medicine, King Abdulaziz Universit, Jeddah 21589, Saudi Arabia; mwalrabia@kau.edu.sa; 5 Department of Natural Products and Alternative, Medicine, Faculty of Pharmacy, King Abdulaziz University, Jeddah 21589, Saudi Arabia; asirwi@kau.edu.sa (A.S.); melfaky@kau.edu.sa (M.A.E.); 6 Department of Medical Laboratory Technology, Faculty of Applied Medical Sciences, King Fahd Medical Research Center, King Abdulaziz University, Jeddah 21589, Saudi Arabia; hsadoun@kau.edu.sa; 7 Department of Clinical Biochemistry, Faculty of Medicine, King Abdulaziz University, Jeddah 21589, Saudi Arabia; beldakhakhny@kau.edu.sa; 8 Department of Biochemistry, Faculty of Science, Cancer and Mutagenesis Unit, King Fahd Medical Research Center, King Abdulaziz University, Jeddah 21589, Saudi Arabia; whabdulaal@kau.edu.sa; 9 Department of Pharmaceutics and Industrial Pharmacy, Faculty of Pharmacy, Cairo University, Cairo 11562, Egypt

**Keywords:** luliconazole, spanlastics, particle size, *Candida albicans* infections, lesion score

## Abstract

Luliconazole is a new topical imidazole antifungal drug for the treatment of skin infections. It has low solubility and poor skin penetration which limits its therapeutic applications. In order to improve its therapeutic efficacy, spanlastics nanoformulation was developed and optimized using a combined mixture-process variable design (CMPV). The optimized formulation was converted into a hydrogel formula to enhance skin penetration and increase the efficacy in experimental cutaneous *Candida albicans* infections in Swiss mice wounds. The optimized formulation was generated at percentages of Span and Tween of 48% and 52%, respectively, and a sonication time of 6.6 min. The software predicted that the proposed formulation would achieve a particle size of 50 nm with a desirability of 0.997. The entrapment of luliconazole within the spanlastics carrier showed significant (*p* < 0.0001) antifungal efficacy in the immunocompromised Candida-infected Swiss mice without causing any irritation, when compared to the luliconazole treated groups. The microscopic observation showed almost complete removal of the fungal colonies on the skin of the infected animals (0.2 ± 0.05 log CFU), whereas the control animals had 0.2 ± 0.05 log CFU. Therefore, luliconazole spanlastics could be an effective formulation with improved topical delivery for antifungal activity against *C. albicans*.

## 1. Introduction

Luliconazole is a new topical imidazole antifungal that belongs to the azoles group with broad-spectrum antifungal activity against pathogenic fungi [1]. It is used as a treatment for superficial infections such as dermatophytosis and candidiasis by inhibiting the ability of fungi to grow and reproduce [2]. It was invented at the Research Center at Nihon Nohyaku Co. Ltd. (Osaka, Japan) then approved in Japan in 2005 as a topical agent [3]. It has lately been approved by the U.S. Food and Drug Administration [4]. It has a minor aqueous solubility which lessens its dermal availability and acts as a hurdle for topical delivery [5]. The most prevalent cutaneous infections by Candida are superficial infections of skin and mucous membranes [6]. It occurs in skin folds, the genitals, cuticles, oral mucosa, or any other part of the body. The signs and symptoms are dependent on the site of infection. Cutaneous infections must be treated by drying and antifungal agents [7].

Although acquired resistance is less common than intrinsic resistance, many studies suggest that it is beginning to emerge for many antifungal drugs in some countries. For example, many studies have reported the ability of *Candida albicans* to develop resistance to fluconazole [8,9]. Oxman and colleagues [8] found that 19% of their Candida infections comprised either fluconazole resistant strains or strains with impaired susceptibility in their recent retrospective case-comparator study undertaken at two tertiary-care cancer centres in Boston, MA, USA. *C. albicans*, *C. tropicalis*, and *C. parapsilosis*, which are considered to be fluconazole sensitive, accounted for 36% of reduced susceptibility isolates and 48% of resistant isolates. Resistance identified in this species may be due to the presence of ERG11 point mutations [10], overexpression of ERG11 [11], and the overexpression of drug efflux pumps [12].

Recently, various topically applied nanocarrier systems have been developed, including lipid based nanocarriers and polymer based nanocarriers, due to their unique advantages and great versatility as compared to conventional formulations [13,14,15,16,17]. In one of the studies, a nanosponge system was found to confine the drug into the pores of this system that showed a good availability of drugs, enhanced skin permeability and extended retention time at the site of application [5]. As well, they found that making the drug in a gel form could present a synergistic effect of extending the retention time due to the high viscosity of this formulation. One more study showed that luliconazole-loaded nanostructured lipid carrier formulations, including lipids and span as a surfactant, had been prepared that indicated better skin penetration, increased retention time and prevented systemic toxicity [18]. Ksur and coworkers developed elastic lipogel and ethogel formulations of luliconazole which included sodium deoxycholate and Tween 80 as an edge activator, in addition to soya phosphatidylcholine as phospholipid and ethanol were found to be more effective against dermatophytes in comparison with the approved formulation [19].

The spanlastics method, which is a new drug delivery system that would directly target the infected cells with minor side effects, works by encapsulating the drug in a vesicle made by a nonionic surfactant that acts as a carrier of the drug to deliver it to the target site. In addition, this nonionic surfactant has good compatibility with biological systems and represents low toxicity. The elastic vesicles refer to the existence of edge activators in their structure [20]. Therefore, the objectives of the study were to prepare and optimize luliconazole spanlastics as potential carriers for topical delivery, using a combined mixture-process variable design (CMPV). Luliconazole spanlastics were prepared which were later converted into hydrogels. The optimized luliconazole spanlastics were evaluated for the experimental cutaneous *C. albicans* infections in Swiss mice wounds.

## 2. Materials and Methods

### 2.1. Materials

Luliconazole was procured as a gift sample from Jamjoom Pharmaceutical, Jeddah, Saudi Arabia. Span 20 and Tween 20 were purchased from Sigma-Aldrich (St. Louis, MO, USA). All other chemicals and solvents were of analytical grade.

### 2.2. Experimental Design

Combined mixture-process variable design (CMPV) was employed for the formulation and optimization of Luliconazole spanlastics. The design was chosen based on its ability to evaluate how the responses are affected by the mixture elements and the process variables simultaneously. In this study, the mixture was composed of two mixture components, namely Span 20 (A) and Tween 20 (B); both were used in percentages ranging from 10–90% so that the total mixture added up to 100%. Sonication time (C) was investigated as process variable (PV) in the range of 0–10 min. The remaining process parameters were kept unchanged in all experimental runs. Particle size (PS, nm) (Y) was considered as a response. The investigated variables with their investigated ranges, in addition to the response and the constraints of the optimization process are compiled in Table 1. Design Expert software (Version 11.0, Stat- Ease Inc., Minneapolis, MN, USA) was applied for the design points generation and statistical analysis of the data obtained. The selection of the design points was based on the D-optimal design where the total runs were 17 and included required model points, lack of fit points, replicate points and additional center points, Table 2.

### 2.3. Preparation of Luliconazole Spanlastics

Seventeen formulations of spanlastics named as F1–F17 were developed using different percentages of Span 20 and Tween 20 as per the CMPV design using a previously reported method [21]. The drug was kept constant at 20 mg in each formulation. The drug and specified amount of Span were dissolved in 5 mL of ethanol, while Tween as an edge activator was dissolved in 10 mL of distilled water at a temperature of 65 °C. The alcoholic solution was injected dropwise into the aqueous solution that was stirred on a magnetic stirrer at a speed of 1000 rpm. The final mixture was kept on the stirrer for an additional 30 min at room temperature. The formed dispersion was then subjected to ultrasonication for the time specified in the design.

### 2.4. Particle Size Measurement

For particle size determination, the dispersions were diluted appropriately with distilled water and then particle size was measured using Zetasizer (Malvern Panalytical Ltd., Malvern, UK) particle size cells. Each sample was measured in triplicate.

### 2.5. Optimization of Luliconazole Spanlastics

The optimized levels for the mixture components and the sonication time were predicted by applying the numerical optimization technique based on desirability approach.

### 2.6. TEM Investigation of the Optimized Luliconazole Splanlastics Formula

The optimized formula dispersion (one drop) was spread on a carbon grid and then phosphotungstic acid was utilized for staining. After that, the sample was dried, and then investigated by TEM (JEM-1011: JEOL, Tokyo, Japan).

### 2.7. Assessment of Antifungal Activity of the Optimized Luliconazole Spanlastics

#### 2.7.1. In Vitro Antifungal Susceptibility Testing

Determination of MIC of Luliconazle and Luliconazole spanlastics against *C. albicans* isolates were conducted in accordance with Clinical Laboratory Standards Institute guidelines using broth microdilution method. Isolates were tested in triplicate and the MIC mode was determined.

#### 2.7.2. Animals

Male adult animals (Swiss mice) weighing 25–30 g were obtained from the animal house of the Faculty of Pharmacy, King Abdulaziz University, Jeddah, Saudi Arabia. The in vivo study protocol was approved by the Animal Ethics Committee of the Faculty of Pharmacy, King Abdulaziz University, Jeddah, Saudi Arabia, ethical approval no. PH-127-41 (2021), in adherence with the Declaration of Helsinki, the Guiding Principle in Care and Use of Animals (DHEW production NIH 80-23) and the Standards of Laboratory Animal Care (NIH distribution #85-23, reconsidered in 1985). Animals were adapted for at least 2 weeks in naturally controlled enclosures (20 ± 1 °C and a 12/12-h dark/light cycle) and were fed pelleted food and tap water ad libitum.

#### 2.7.3. Candida and Culture Conditions

*C. albicans* (ATCC 90028) was kept on Sabouraud’s dextrose agar (SDA) plate for 48 h at 35 °C. Colonies were suspended in 5 mL 0.85% sterile phosphate buffer saline (PBS). The final concentration was adjusted to 2 × 10^7^ CFU/mL.

#### 2.7.4. Animal Preparation and Cutaneous Infections

Twenty adult Swiss mice were randomly divided into four groups (*n* = 5/group). Mice were intraperitoneally injected by cyclophosphamide (100 mg/kg/day) for three days prior to fungal infection to induce immunocompromised animals [22].

Induction of cutaneous candidiasis model was made following Maebashi et al. [2] with some modification. The backs of the mice were shaved with an electronic shaver (area 2 × 2 cm). After 48 h, the skin was moderately abraded with sandpaper. One hundred microliters of Candida cell suspension (2 × 10^7^ cells) were gently applied by cotton-tipped swab onto the skin. 

#### 2.7.5. Treatment of the Infection

Dosing was giving once a day for five consecutive days, starting 24 h after Candida infection. Group 1 was negative control with no infection and no treatment (control group), group 2 was positive control receiving infection with no treatment (untreated group), group 3 applied topically with Luliconazole 25 mg/kg/day (Luli group), and group 4 applied topically with equivalent dose of Luliconazole spanlastics 25 mg/kg/day (Luli-span group). 

#### 2.7.6. Evaluation of Infection

Macroscopic evaluation of infection was measured by a score of erythema from 0 to 4 as described (2): 0, not erythematous (normal); 1, slightly erythematous; 2, moderately erythematous; 3, spreading erythematous; and 4, severely erythematous.

For microbiological evaluation of infection, mice were sacrificed 24 h following the last dose and 1 × 1 cm of skin from the infected sites was excised. The infected skin samples were washed with sterile PBS and plated onto SDA plates then incubated for 48 h at 37 ± 1 °C, and CFU values of *C. albicans* were recorded. 

Data were presented as mean ± standard error and were statistically analyzed using one-way ANOVA (SPSS, Inc., Chicago, IL, USA) to measure the differences between the parameters. The confidence level using GraphPad Prism 6 (GraphPad Software, San Diego, CA, USA) was set at * *p* < 0.01 and ** *p* < 0.001.

## 3. Results and Discussion

### 3.1. Particle Size Results and Model Fit Statistical Analysis

The variables’ levels for the luliconazole spanlastics runs and the measured particle size for each run are displayed in Table 2. The mean particle size exhibited a marked variation ranging from 60.8 to 5891 nm. The fit statistics analysis was carried out to produce a CMPV polynomial model illustrating the relation between the particle size and the studied MCs and PV. The statistical software suggested the quadratic × cubic (Q × C) based on the highest adjusted R^2^ (0.9436). In addition, adequate precision of 18.05 (greater than 4) indicated appropriate signal to noise ratio [23]. Accordingly, the suggested model could be applied to navigate the experimental space. The polynomial equation that describes the particle size in terms of L-Pseudo components of the mixture and coded factor for the sonication time was developed by the software as follows:

Y = 222.28 A + 260.82 B − 281.94 AB − 553.32 AC − 1804.21 BC + 4940.31 ABC + 880.84 AC^2^ + 2088.93 BC^2^ + 19,106.27 AB(A − B) − 6088.71 ABC^2^ − 4231.70 ABC(A − B) − 71,146.97 ABC^2^(A − B)

The equation in terms of coded factors can be utilized for predicting the response for given levels of each factor. The high levels of the mixture components and process factors were coded as +1, the low levels of the mixture components were coded as 0, and the low levels of the process factors were coded as −1. The coded equation is advantageous for finding the relative influence of the factors by comparing the corresponding coefficients. 

The presence of significant MPV coefficients in the equations highlights the usefulness of employing the CMPV design as it reveals the interaction between the MCs and the PV; such interaction could never be detected using a traditional one factor at a time approach or even experimental designs done individually on MCs and PVs [24,25].

### 3.2. Diagnostics for the Validity of the Quadratic Model

A diagnostic plot of externally studentized residuals versus run for particle size was generated to establish the goodness of fit of the quadratic model. Figure 1 displays randomly distributed points showing that no lurking variable could influence the measured response [15,26].

### 3.3. Influence of Variables on Particle Size (PS, Y*_1_*) 

Reducing the particle size of the vesicular systems to the nano-range could markedly contribute to promoting the absorption of active ingredients and/or improving their biological performance [27]. The Q × C model was significant for the particle size data (*p* = 0.0011). The computed F-values of 25.23 confirmed the significance of the model; there was only a chance of 0.11% that such a value could be this large owing to noise. Lack of fit F-values of 0.37 showed a nonsignificant lack of fit in relation to the pure error indicating fitting of the data to the model. According to the computed *p*-values, the terms AC, BC, ABC, BC^2^, AB(A − B), ABC^2^, ABC^2^(A − B) were significant (*p* < 0.05) on the measured data. The three-dimensional mixture-process plot for the particle size are presented in Figure 2. 

### 3.4. Optimization Using a Numerical Approach

The aim of optimization in the formulation field is to predict the values of the variables that could yield a product with the desired characteristics. In our study, the optimization process aims at obtaining Luliconazole spanlastics with minimized particle size. The numerical optimization technique was adopted to achieve this aim. The optimized formulation was generated at percentages of Span and Tween of 48% and 52%, respectively, and a sonication time of 6.6 min. The software predicted that the proposed formulation could achieve a globule size of 50 nm with a desirability of 0.997.

### 3.5. Transmission Electron Microscope Investigation of the Optimized Luliconazole Spanlastics

Transmission electron microscope (TEM) photographs of the optimized formula showed rounded structures which revealed some aggregations that could be attributed to the process of drying during sample preparation (Figure 3).

### 3.6. In Vitro Antifungal Susceptibility Testing

An in vitro antifungal susceptibility study using broth microdilution was carried out where the minimum inhibitory concentrations (MIC) of the luliconazole spanlastics were compared with those of luliconazole alone against *C. albicans* (ATCC 90028). Results revealed no differences in the susceptibility patterns between the tested components.

### 3.7. In Vivo Study

Being the most opportunistic pathogen for human infection, *C. albicans* are known to invade superficially and simultaneously spread fungal infection. Furthermore, the growing emergence of developing resistance by the fungal species and the unfavorable outcomes of the conventional treatments urges novel deliveries [28]. Five days consecutive cutaneous treatment of the immunocompromised animals with Candida infection showed promising results as depicted in Figure 4 and Figure 5.

The animals in Group 1 did not show any signs of infection as clearly shown in Figure 4A,B, whereas the average lesion score of the infected animals was demonstrated to decrease with the days of treatments. As there was no treatment provided to the infected animals in Group 2, the rate of subsiding of the infection in those animals is much less. On the other hand, treatment of the infected animals with luliconazole was found to decrease the average lesion score of the animals in Group 3 (Figure 4A,B). Our findings on the obtained antifungal efficacy of luliconazole (25 mg/kg/day) showed agreement with the existing literature where the control of bacterial infection using luliconazole was equivalent [29]. Furthermore, treatment of luliconazole spanlastics to the animals in group 4 showed outstanding control of infections as depicted by the significant (*p* < 0.0001) reduction in the lesion score with significant reduction in the erythema score when compared to the results obtained in Group 3, treated with luliconazole (Figure 3 and Figure 4). This significant recovery of the animals was clearly demonstrated in Figure 4, where the gradual recovery of the experimental animals administered with luliconazole spanlastics is clearly displayed. This superior efficacy of the drug (luliconazole) using a spanlastics platform over the plain luliconazole treatment might be explained by the preeminence in topical delivery of luliconazole-loaded surfactant-based elastic nanovesicles [30].

Furthermore, the inoculation of *C. albicans* to the abraded skin of the animals showed white patches composed of microscopic colonies when observed under microscope. There were no colonies observed in the control group, whereas the number of colonies in the untreated animals after five days of inoculation was recorded as 14 ± 2.2 log CFU at the infected site (Table 3). This number was found to be decreased significantly (*p* < 0.0001) in the luliconazole treated animals when compared to the untreated animal groups. Moreover, the log colonies in the animals of the luliconazole spanlastics treatment group was found to 0.2 ± 0.05, which is statistically significant (*p* < 0.0001) when compared to the results of luliconazole treatment group. Thus, the microscopic findings of the animals treated with the spanlastics delivery is comparable to the macroscopic findings of the animal skin.

## 4. Conclusions

The luliconazole spanlastics were prepared and optimized based on three factors, i.e., the ratio of Tween 20, Span 20 and sonication time. The software predicted that the proposed formulation would achieve a particle size of 50 nm with a desirability of 0.997. The optimized spanlastics showed increased topical delivery for a drug with poor aqueous solubility. In vivo antifungal efficacy in experimental Swiss albino mice represented extraordinary results in controlling the Candida infection in experimental animals. This improved control in the removal of fungal colonies from the infected skins of immunocompromised animals might be because of improved permeation of the drug through this vesicular delivery system. In conclusion, luliconazole spanlastics could be an effective formulation with improved topical delivery for antifungal activity against *C. albicans*.

## Figures and Tables

**Figure 1:** Externally studentized residuals vs. run number for the quadratic × cubic model for luliconazole spanlastics particle size.

**Figure 2:** Effect of the binary mixture components (I) and the sonication time (II) at the mid-values of the other variables; Three-dimensional mixture−process plot (III) for the particle size of luliconazole spanlastics.

**Figure 3:** Transmission electron microscope photograph of optimized luliconazole spanlastics.

**Figure 4:** Establishment of infection expressed as lesion score after starting treatment in cutaneous candidiasis mouse model. Mice (*n* = 5/group) were applied topically with luliconazole 25 mg/kg/day as Luli group and equivalent dose of luliconazole spanlastics (Luli-span group) for 5 days. (**A**) The score of erythema were measured on days 1, 3 and 5. (**B**) Average lesion score in *C. albicans* induced cutaneous candidiasis in mice treated with different formulations and compared with control and untreated group on the 5th day. Data were presented as mean ± SD. @ significant Luli span vs. untreated (*p* < 0.0001). * Significant Luli span vs. Luli group (*p* < 0.0001) determined by student *t* test.

**Figure 5:** Macroscopic evaluation of infection was measured by a score of erythema in mice of all three groups at 1, 3 and 5 days. On the 1st day after induction of *C. albicans* cutaneous candidiasis, obvious infection developed in all groups. On 3rd day small recovery was observed in luliconazole (Luli group) and luliconazole spanlastics (Luli-span group). On 5th day significant recovery was observed in Luli-span group.

**Table 1:** Ranges of mixture components and process variables and the desired constraints of the response variables for the CMPV design.

Mixture Components	Lower Level	Upper Level
A: Span 20 percentage	10	90
B: Tween 20 percentage	10	90
**Process Variable**		
C: Sonication time (min)	0	10
**Responses**	**Desirability Constraints**	
Y: Particle size (PS, nm)	Minimize	

Abbreviations: CMPV, combined mixture process variable.

**Table 2:** The variables’ levels and the observed responses of luliconazole spanlastics runs.

Run No.	Mixture Components		Process Variables	Particle Size (nm)
	A	B	C	
1	90	10	10	307.6
2	10	90	10	701.9
3	50	50	0	198.0
4	10	90	5	256.2
5	30	70	2.5	166.1
6	30	70	7.5	330.7
7	90	10	0	1204.0
8	10	90	0	4174.0
9	70	30	7.5	324.1
10	90	10	0	2130.0
11	70	30	2.5	327.5
12	90	10	10	771.5
13	10	90	10	367.6
14	30	70	0	5891.0
15	90	10	5	218.2
16	50	50	10	60.8
17	50	50	5	143.6

Abbreviations: A, Span percentage; B, Tween percentage; C, sonication time (min).

**Table 3:** Colony-forming units of *C. albicans* on the skin of mice after treatment with different formulations.

Sample No.	Treatment (groups)	Number of Animals	Log CFU Infected Site
1	Control	5	0
2	Untreated	5	14 ± 2.2
3	Luliconazole	5	3.1 ± 0.2
4	Luliconazole spanlastics	5	0.2 ± 0.05 *

Values represent mean ± SD. * Significant reduction in fungal count of Luliconazole spanlastics versus Luliconazole treatment (* *p* < 0.001) determined by Student’s *t* test.

## Data Availability

Data are available within the manuscript.
